The article "Optimization of Correlation Filters Using Extended Particle Swarm Optimization Technique" was retracted in 2023. Reasons: unreliable results or conclusions; concerns about the data; concerns about the peer review; concerns about the citations.

# Optimization of Correlation Filters Using Extended Particle Swarm Optimization Technique

**DOI:** 10.1155/2021/6321860

**Published:** 2021-07-05

**Authors:** Haris Masood, Amad Zafar, Muhammad Umair Ali, Muhammad Attique Khan, Kashif Iqbal, Usman Tariq, Seifedine Kadry

**Affiliations:** ^1^Wah Engineering College, University of Wah, Wah Cantt, Pakistan; ^2^Department of Electrical Engineering, University of Lahore, Islamabad Campus, Pakistan; ^3^Department of Unmanned Vehicle Engineering, Sejong University, Seoul 05006, Republic of Korea; ^4^Department of Computer Science, HITEC University Taxila, Taxila 47040, Pakistan; ^5^College of Computer Engineering and Sciences, Prince Sattam Bin Abdulaziz University, Al-Khraj, Saudi Arabia; ^6^Faculty of Applied Computing and Technology, Noroff University College, Kristiansand, Norway

## Abstract

In the past few decades, the field of image processing has seen a rapid advancement in the correlation filters, which serves as a very promising tool for object detection and recognition. Mostly, complex filter equations are used for deriving the correlation filters, leading to a filter solution in a closed loop. Selection of optimal tradeoff (OT) parameters is crucial for the effectiveness of correlation filters. This paper proposes extended particle swarm optimization (EPSO) technique for the optimal selection of OT parameters. The optimal solution is proposed based on two cost functions. The best result for each target is obtained by applying the optimization technique separately. The obtained results are compared with the conventional particle swarm optimization method for various test images belonging from different state-of-the-art datasets. The obtained results depict the performance of filters improved significantly using the proposed optimization method.

## 1. Introduction

For the purpose of object detection and recognition in the fields of pattern recognition, computer vision, and image processing [1–5], correlation filters have been widely employed. Other fields in which correlation filters are used are object tracking [6, 7] and biometric object recognition [8–10]. The correlation filters are trained in a way to generate maximum correlation peaks pertaining to the objects desirous of being detected, while generation low peaks against illumination, clutter, and noise. Correlation filters date back to around three decades, when they were introduced primarily for object recognition [11]. Over the years, improvement in the accuracy of the correlation filters has been made, using different optimization methods [12–15].

Accurate recognition and tracking of objects can be carried out using the correlation filters. The Maximum Average Correlation Height (MACH) and Maximum Average Correlation Energy (MACE) are used for eliminating clutter distortion and noise [16]. The MACE filter is extremely sensitive to clutter and noise, while providing distinct peaks for the detection of filter outputs [17]. The MACH filter gives maximum relative height w.r.t the expected distortions by generating the broader peaks [18].

The article "Optimization of Correlation Filters Using Extended Particle Swarm Optimization Technique" was retracted in 2023. Reasons: unreliable results or conclusions; concerns about the data; concerns about the peer review; concerns about the citations.

Complex filter equations are employed for implementing the correlation filters in different software. Thus far, many correlation filters' variants have been introduced by altering values of the optimal tradeoff (OT) parameters of involved filter equations. Up till now, experimental trials have been conducted for tuning of the tradeoff parameters. The main motivation of the proposed research is to optimize the OT parameters using a technique that has not been employed before, which enables determining the best possible values. The optimization technique presented in this paper is based on the particle swarm optimization (PSO) variant. The PSO algorithm was first introduced by Eberhart and Kennedy [19]. It is a population-oriented method that is inspired by animals and fish social behavior. The standard PSO algorithm [20] is the one used for basic optimization of parameters. EPSO proposed by Li et al. [21] is considered to be PSO's most renowned variant. This particular variant has been employed in various applications of image processing [22–28].

The paper compares the standard PSO and EPSO for OT parameter optimization. The parametric optimization relies on MACH and MACE filter cost functions. The filters produced as a result are application specific as the parameter values vary based on each target object of interest. The filter is generic in nature as given the application, it can be applied successfully on any target object of interest based on calculations of the cost functions. The proposed algorithm is novel in the sense that PSO variants have not been previously employed in conjunction with correlation filters for accurate object recognition. Previously, values suggested by Bone et al. were used for the optimization of optimal tradeoff values of a correlation filter. This is the first time that an ensemble of EPSO and correlation filters is used for the optimization of optimal tradeoff parameters for accurate object detection.

## 2. Proposed Methodology

### 2.1. Correlation Filters

The main motivation behind employing the enhanced version of the correlation filter is to exclude the peaks that make the procedure of object detection, an erroneous one. In multiplexed filters, it is usually very difficult to obtain a sharp peak using the correlation templates, which often outputs high-intensity side lobes. For easy detection of object of interest, MACE filters are employed, which are responsible for providing sharp peaks. The downside of MACE filters is that they are sensitive to distortion. In the MACE filter, the function level is evenly reduced over the entire correlation plane, with the exception of the plane center. On the contrary, MACH provides broader correlation peaks, but it comes with an added advantage of being noise and distortion tolerant. For the implementation of MACE and MACH filters, the metrics of Average Correlation Energy (ACE) and Average Similarity Matrix (ASM) are minimized, respectively. Since minimization of ASM is directly related to the reduction of dissimilarity among the correlation planes, it makes the correlation process more accurate. The amplitude of peaks of the MACH filter is higher than the MACE filter peaks [17, 18].

The article "Optimization of Correlation Filters Using Extended Particle Swarm Optimization Technique" was retracted in 2023. Reasons: unreliable results or conclusions; concerns about the data; concerns about the peer review; concerns about the citations.

Equation (1) shows the energy equation [29] pertaining to the correlation filter.

(1) $$\begin{array}{c} E\left(f\right)=\alpha \left(\text{ONV}\right)+\beta \left(\text{ACE}\right)+\gamma \left(\text{ASM}\right)-\delta \left(\text{ACH}\right). \end{array}$$

The ASM can be calculated using

(2) $$\begin{array}{c} \text{ASM}=f^{+}S_{x}f, \end{array}$$

(3) $$\begin{array}{c} S_{x}=\frac{1}{N}\overset{N}{\underset{i=1}{\sum }}{\left(X_{i}-M_{x}\right)}^{*}\left(X_{i}-M_{x}\right), \end{array}$$

where the variable “*f*” depicts the chosen filter and the “+” sign in the superscript depicts the conjugate response in Equation (2).

The ACE of the filter can be computed using

(4) $$\begin{array}{c} \text{ACE}=f^{+}D_{x}f,\\ D_{x}=\frac{1}{N}\overset{N}{\underset{i=1}{\sum }}X_{i}^{*}X_{i}. \end{array}$$

Equation (5) is used for the calculation of output noise variance [9].

(5) $$\begin{array}{c} \text{ONV}=f^{+}Cf. \end{array}$$

The variable “*C*” indicates a diagonal *d*∗*d* dimensional vector. Normally, the value of *C* is taken as *δ*^2^*I*. Equation (6) is used for the calculation of Average Correlation Height (ACH) [29].

(6) $$\begin{array}{c} \text{ACH}=\left|\frac{1}{N}\overset{N}{\underset{i=1}{\sum }}f^{T}X_{i}\right|=\left|f^{T}m_{x}\right|, \end{array}$$

where *m*_*x*_ represents the average of *N* vectors.

By substituting all the values, Equation (1) can be minimized into

(7) $$\begin{array}{c} E\left(f\right)=f^{+}\text{If}-\delta \left|f^{T}m_{x}\right|, \end{array}$$

where *I* can be described using

(8) $$\begin{array}{c} I=\alpha C+\beta D_{x}+\gamma S_{x}. \end{array}$$

Therefore, the filter equation becomes

(9) $$\begin{array}{c} f^{o}=\left(\frac{\delta }{2}\right)I^{-1}m_{x}, \end{array}$$

where *δ* represents the scaling factor and *o* in the superscript depicts optimal complex filter transfer function. The values of *α*, *β*, and *γ* are nonnegative entities. The effectiveness of the MACH filter depends mainly on the adjustment of these three parameters, i.e., *α*, *β*, and *γ*. By selecting *α* = 0 and *γ* = 0, the filter transfer function is transformed into a simple MACE filter which is used for the minimization of ACE. Setting *α* = 0 and *β* = 0 converts the filter transfer function to the MACH filter which is used for the minimization of ASM. Up till now, the optimized values as suggested by Bone et al. have been kept at *α* = 0.01, *β* = 0.1, and *γ* = 0.3, since they are considered optimal for the implementation of the MACH filter. In reality, these values do not show promising results for some datasets as the conditions in different scenarios vary. In this paper, a novel method using EPSO has been proposed for calculating the optimal OT values that can be considered optimal for every environment.

The article "Optimization of Correlation Filters Using Extended Particle Swarm Optimization Technique" was retracted in 2023. Reasons: unreliable results or conclusions; concerns about the data; concerns about the peer review; concerns about the citations.

A combination of a correlation filter and an optimization technique is proposed in this paper. The combined optimized filter provides optimal values of OT parameters based on the specific target object of interest. The results of conventional PSO and proposed EPSO algorithms will be compared in the later section of the paper.

### 2.2. Particle Swarm Optimization

PSO, as previously described, is an optimization algorithm that is derived from fish schooling and motion of bird flocks. PSO is a very good technique used primarily for the optimization of the parameters. PSO searches the most optimal solution in a multidimensional search space with the help of several available particles who all donate towards the optimized particles. The algorithm searches the best value for each particle by the convergence method. A cost function is employed for the estimation of each optimized value. The cost function is also used to identify the most suitable value for the defined fitness function. Two primary parameters are associated with each particle: (i) the velocity of each particle *v*(*i*) and (ii) the particle position of each particle *x*(*i*), where the iteration index is indicated by *i*. Subsequently, the global best of whole swarm is obtained by extracting the best values related to all the particles and combining them. In a *D*-dimensional space involving a swarm of *N* particles, the position and velocity of each particle are updated using

(10) $$\begin{array}{c} v_{k}^{d}\left(i+1\right)=w.v_{k}^{d}\left(i\right)+c_{1}.r_{1,k}\left(i\right).\left(p_{k}^{d}-x_{k}^{d}\left(i\right)\right)+c_{2}.r_{2,k}\left(i\right).\left(g^{d}-x_{k}^{d}\left(i\right)\right), \end{array}$$

(11) $$\begin{array}{c} x_{k}^{d}\left(i+1\right)=x_{k}^{d}\left(i\right)+v_{k}^{d}\left(i+1\right), \end{array}$$

where the dimensions of the particles are denoted by *d* = 1, 2 ⋯ , *D* and the particle index is denoted by *k* = 1, 2 ⋯ , *N*. The constants *c*_1_ and *c*_2_ represent the cognitive and social coefficients, respectively. The velocity and position of the *k*th particle are represented by *v*_*d*_^*k*^ and *x*_*d*_^*k*^, respectively, in a *d*-dimensional space. The particles' local best position is represented by *p*_*d*_^*k*^, while *g*_*d*_ represents the swarms' global best position. While searching the behavior of the swarm, the source of randomness and uniform random distribution [0, 1] are the two parameters used for the derivation of *r*_1,*k*_ and *r*_2,*k*_.

The article "Optimization of Correlation Filters Using Extended Particle Swarm Optimization Technique" was retracted in 2023. Reasons: unreliable results or conclusions; concerns about the data; concerns about the peer review; concerns about the citations.

The most popular variant of the PSO was proposed by Eberhart and Kennedy. Equation (12) shows the variant that contains a model based on inertial weight [19]. The model tends to multiply a constant factor commonly known as the weight of the inertia, with the velocity of the current iteration [19].

(12) $$\begin{array}{c} v_{k}^{d}\left(i+1\right)=w.v_{k}^{d}\left(i\right)+c_{1}.r_{1,k}\left(i\right).\left(p_{k}^{d}-x_{k}^{d}\left(i\right)\right)+c_{2}.r_{2,k}\left(i\right).\left(g^{d}-x_{k}^{d}\left(i\right)\right). \end{array}$$

The momentum of the particle is controlled by the convergence of inertia weight *w* *ϵ* [0, 1]. For a small value of *w*, negligible momentum is preserved and carried forward from the previous iteration that tends to change the direction quickly. On the contrary, a larger *w* value means slow convergence and delayed change in particle direction. For the value of *w* = 0, the particle moves ahead without any prior knowledge of the value of velocity. The defined variant is commonly known as the standard PSO [30, 31].

The optimization algorithms have several applications associated with them. Pandey et al. [32] employed the PSO algorithm for clustering of data vectors. The algorithm was also used for the user-defined centroid of data clusters and their identification. While comparing PSO with its counterpart, i.e., the *k*-means clustering technique, the PSO returned the best convergence with minimal errors. The proposed PSO algorithm by Nayyar et al. is now used in conjunction with *k*-means for the refinement of clusters [24]. Grosan et al. [33] proposed an application pertaining to the PSO algorithm in data mining domain. They used the PSO algorithm for cloud computing such that applications were efficiently scheduled by optimizing the cloud resources. As compared to the heuristic algorithms, the proposed technique by Grosan et al. reduced the cost of data transmission and computation by one-third. As compared to the *k*-means algorithm, the PSO algorithm for the optimization of image clustering was utilized. Applications can be found in satellite imaging and in MRI as well.

The article "Optimization of Correlation Filters Using Extended Particle Swarm Optimization Technique" was retracted in 2023. Reasons: unreliable results or conclusions; concerns about the data; concerns about the peer review; concerns about the citations.

The most commonly employed PSO variant is the extended PSO having the time-varying coefficients related to acceleration (EPSO) [22]. An optimal solution is obtained through the acceleration coefficients only by guiding the movement of particles, while coefficients related to inertia are removed. The coefficients related to acceleration move linearly with respect to time. Therefore, if at some point, velocity goes to zero, the particle is reinitialized through the use of other predefined velocities.

### 2.3. Extended Particle Swarm Optimization (EPSO) Algorithm

In each iteration of the conventional PSO technique, two extreme values are used for updating the state of each particle. For optimizing the algorithm's global convergence and to increase its efficiency, the global impact of many involved particles contributes towards updating the state of each particle. Such an impact caused by the multiparticle effect is commonly known as the extended particle swarm optimization (EPSO) algorithm.

In EPSO algorithms' recursive process, the optimization process includes particles that contain more information as compared to the conventional PSO. The main formula of EPSO is stated in Equations (13) and (14) [21].

(13) vi+1=wvt+∑i=1mψipt−xt+∑i=1nζip^t−xt,

(14) $$\begin{array}{c} x_{i+1}=x_{t}+v_{t+1}, \end{array}$$

where *ψ*_*i*_ = *c*_1,*i*_*r*_1,*i*_(0, 1) and *ζ*_*i*_ = *c*_2,*i*_*r*_2,*i*_(0, 1) [21].

The number of iterations is depicted by the subscript *t*, *v*_*t*_ denotes the velocity of the particles, *x*_*t*_ denotes the interspaces of the involved particles, *p*_*t*_ signifies the extreme value particle's position, p^t denotes the local extreme particles, and *r*_1,*I*_ (0, 1) and *r*_2,*I*_ (0, 1) are random variables between 0 and 1, while *c*_1,*I*_ and *c*_2,*i*_ represent the control parameters. A comparison of Equations (14) and (12) shows that in comparison with the conventional PSO, EPSO takes into account the information associated with more particles involved in the optimization process, thus providing stronger and better global convergence. EPSO can easily be converted to the conventional PSO by setting values of *m* = *n* = 1.

Since the EPSO utilizes information from more particle values and it also considers more particles and more controlled parameters for the optimization process, the parameter selection has to be spot on in order for the algorithm to converge quickly. The setting strategy pertaining to the control parameters of the algorithm is obtained by testing the convergence condition of the EPSO algorithm. The iterative formula for the EPSO algorithm is calculated by substituting Equation (13) in Equation (14) and using *v*_*t*_ = *x*_*t*_ − *x*_*t*−1_. Equation (15) describes the main cumulative formula [21].

(15) xi+1=1+w−∑i=1mψi+∑i=1nζixt−wxt−1+∑i=1mψipi+∑i=1nζipt^.

The article "Optimization of Correlation Filters Using Extended Particle Swarm Optimization Technique" was retracted in 2023. Reasons: unreliable results or conclusions; concerns about the data; concerns about the peer review; concerns about the citations.

Since for all the iterations, *p*_*t*_ and p^t are considered constants, therefore, Equation (15) can be summarized to Equation (16) [21].

(16) $$\begin{array}{c} \left[\begin{array}{c} x_{t+1}\\ x_{t}\\ 1 \end{array}\right]=\left[\begin{array}{ccc} 1+w-\psi -\zeta & -w & \psi p+\zeta p\\ 1 & 0 & 0\\ 0 & 0 & 1 \end{array}\right]\left[\begin{array}{c} x_{t}\\ x_{t+1}\\ 1 \end{array}\right], \end{array}$$

where *ψ* = ∑_*i*=1_^*m*^*ψ*_*i*_, *ζ* = ∑_*i*=1_^*m*^*ζ*_*i*_, *ψp* = ∑_*i*=1_^*m*^*ψ*_*i*_*p*_*t*_, and ζp=∑i=1nζip^t [21].

The velocity solution is obtained by generalizing Equation (13), and Equation (14) can be categorized into Equation (17) [22].

(17) $$\begin{array}{c} v_{k}^{d}\left(i+1\right)=c_{1}.r_{1,k}\left(i\right).\left(p_{k}^{d}-x_{k}^{d}\left(i\right)\right)+c_{2}.r_{2,k}\left(i\right).\left(g_{d}-x_{k}^{d}\left(i\right)\right), \end{array}$$

where [22]

(18) $$\begin{array}{c} c_{1}=\left(c_{1f}-c_{1i}\right)*\frac{k}{\max\text{ITER}}+c_{1i},\\ c_{2}=\left(c_{2f}-c_{2i}\right)*\frac{k}{\max\text{ITER}}+c_{2i}. \end{array}$$

Recursive updating of the position and velocity of the *k*th particle is carried out using Equations (16) and (17), respectively.

### 2.4. EPSO for Designing of Correlation Filter

Implementation of correlation filters is performed using complex filter transfer functions which are dependent on the selection of tradeoff parameters. The tradeoff parameters should be optimal in order for the filter to work in an effective manner. Better selection of tradeoff parameters will result in accurate correlation peaks and thus better object detection. Several researchers have proposed methods for the effective calculation of these values. A method proposed by Bone et al. [16] used fixed values for the optimal tradeoff parameters. The choice of selection of these values was not obvious for certain object recognition applications. A novel technique for efficient selection of these tradeoff parameters is proposed in this paper which pertains to the response of the filter. The parameter *α* mentioned in Equation (8) can be calculated using Equation (15) [22].

(19) $$\begin{array}{c} \alpha_{k}\left(t+1\right)=\alpha_{k}\left(t\right)+v_{k,\alpha }\left(t+1\right). \end{array}$$

Similarly, using Equations (15) and (17), similar equations of *β* and *γ* can be obtained for the purpose of optimization. EPSO calculates the values of optimal tradeoff parameters via convergence of the involved fitness function. It will enable the fitness function to be calculated for specific object recognition applications by calculating the correlation output peak intensity (COPI) cost function and peak to correlation energy (PCE) cost function. The correlation pertaining to the object of interest depends on the calculation of COPI and PCE cost functions. The calculation of both of these parameters is performed for the characterization of the correlation plane [34], as mentioned in Equations (20) and (21) [9].

(20) $$\begin{array}{c} \text{COPI}=\max\left\{{\left|C\left(x,y\right)\right|}^{2}\right\}. \end{array}$$

*C*(*x*, *y*) depicts at location (*x*, *y*) the correlation peak output and [9]

(21) $$\begin{array}{c} \text{PCE}=\frac{\text{COPI}-\overset{\_\_\_\_\_\_\_\_\_\_\_\_\_}{{\left|C\left(x,y\right)\right|}^{2}}}{{\left\{\sum \left({\left[{\left|C\left(x,y\right)\right|}^{2}-\overset{¯}{{\left|C\left(x,y\right)\right|}^{2}}\right]}^{2}/\left(N_{x}N_{y}-2\right)\right)\right\}}^{1/2}}, \end{array}$$

where the average COPI is represented by ${\left|\bar{C\left(x\right.,y}\right|}^{2}=\sum {\left|C\left(x\right.,y\right|}^{2}/N_{x}N_{y}$.

The article "Optimization of Correlation Filters Using Extended Particle Swarm Optimization Technique" was retracted in 2023. Reasons: unreliable results or conclusions; concerns about the data; concerns about the peer review; concerns about the citations.

For maximizing the PCE cost function, the value of ACE is reduced by the MACE filter. The MACH filter is responsible for minimizing the ASM value. The height of the correlation peak is maximized due to the reduction of ASM. In the optimization algorithms, fitness functions are defined by COPI and PCE values. The summary of the steps is mentioned in Tables 1 and 2.

## 3. Results and Discussion

Eight publicly available datasets [35, 36] have been used for the experiments and analysis. Five datasets are vehicle-oriented datasets in which the object of interest, i.e., the vehicle, undergoes different shift, scale, occlusion, and lightening conditions. Three remaining datasets, i.e., Singer, Blur Body, and Skating, are person-oriented datasets in which the object of interest, i.e., person, undergoes motion blur, shift, scale, and occlusion-based variations. The obtained results have been used for the comparison of results of the proposed algorithm with other similar state-of-the-art algorithms [16].

### 3.1. Setting of Parameters

In order to test and evaluate the optimal values of tradeoff parameters, experiments have been carried out using both the PSO and EPSO techniques. The chosen parameters are shown in Table 3.

Implementation of parameters has been ensured with a slight modification. Since there is a possibility that particles may give negative values for some particular parameters, only the magnitude is considered, while ignoring the sign. The lower limit of values has been set to -0.1 to give weightage to the lower order negative values. The results proved that the assumption was correct.

The article "Optimization of Correlation Filters Using Extended Particle Swarm Optimization Technique" was retracted in 2023. Reasons: unreliable results or conclusions; concerns about the data; concerns about the peer review; concerns about the citations.

### 3.2. Comparison of Results of PSO and EPSO

Eight publicly available datasets shown in Figure 1 were tested for acquiring the results. The chosen datasets were based on the diversity of the conditions that the images of datasets were taken. The chosen datasets have been employed for comparison of results of the algorithms and analyzing the optimized values of each dataset. The 0-45 training images were rotated out-of-plane. Among the images, a difference of 10 was ensured. Cost function has been chosen based on the requirement in hand. As a cost function, both the COPI and PCE values have been individually selected for comparison of the EPSO and PSO results with the Bone et al. suggested values [16].

Testing images belonging to different datasets and for different rotations are used for the analysis of the optimized values and for experimentation purposes. For the Bone et al. algorithm, the values of *α*, *β*, and *γ* have been set as 0.01, 0.1, and 0.3, respectively, as previously proposed.  Table 4 shows the comparison based on COPI cost function between the proposed values of Bone et al. and the optimized values calculated through the proposed algorithm. The results evidently depict that the correlation peaks generated by the EPSO optimization algorithm are better than the peaks generated by PSO and Bone et al. values.

The optimization algorithms have been employed for the comparison with Bone et al.'s proposed values using one of the proposed datasets from Table 4. As a cost function, the COPI value has been used for the algorithms. Results clearly depict that in comparison with the PSO and Bone et al.'s algorithms, the optimized values from EPSO perform very well considering the COPI cost function as shown in Figure 2. Out of plane rotation of 15° is applied on the testing images. The attained COPI values in the cases of EPSO, PSO, and Bone et al. are 3.24*E* − 2, 5.15*E* − 4, and 7.05*E* − 5, respectively. The peaks obtained from Bone et al. and PSO values are approximately the same as evident in Figures 2(a) and 2(b), respectively. However, the results of applying the PSO far outmatch the results obtained from Bone et al.'s proposed parameter values. The COPI results obtained from using the optimized parameter values of EPSO are far better than the results obtained from both the Bone et al. algorithm and the standard PSO, as shown in Figure 2(c). The EPSO result for other performance metrics is also better than the algorithms proposed by Bone et al. and standard PSO as mentioned in Figures 3–5.  Table 4 also depicts that EPSO outperforms the PSO and Bone et al. algorithm at varying degree levels which shows that the algorithm is shift tolerant. Since all of the eight datasets include images with varying scaling levels, therefore, it is evident from the results depicted in Table 4 that EPSO provides scale invariance as well.

The article "Optimization of Correlation Filters Using Extended Particle Swarm Optimization Technique" was retracted in 2023. Reasons: unreliable results or conclusions; concerns about the data; concerns about the peer review; concerns about the citations.

A testing image that has been rotated out of plane by 45° is shown in Figure 3. The achieved COPI values for EPSO, PSO, and Bone et al. are 3.24*E* − 2, 5.15*E* − 4, and 7.05*E* − 5, respectively. In the correlation plane, the presence of side lobes using optimized values of EPSO is due to the occurrence of ONV as well as due to the inclusion of full correlation process in the experimentation, i.e., full correlation of the testing image is performed with the filter. Considering the COPI cost function, the results of EPSO optimized values outmatch the results of the other values.

The maximum value of the PCE parameter can be achieved by minimizing the ACE value. This leads to a prominent and sharper peak as compared to the other methods. The pattern of optimized values is examined by experimenting on different datasets consisting of test images that have been rotated out of plane. The parameters *α*, *β*, and *γ* have been set as 0.01, 0.1, and 0.3, respectively. The comparison between the proposed algorithm and Bone et al.'s algorithm based on PCE cost function is shown in Table 5. The results evidently show that the PCE values generated by the EPSO optimization algorithm outmatch the values generated by PSO and Bone et al.'s values.

Different datasets have been employed for the analysis of correlation plane based on PCE function. The testing image is rotated out of plane by 45° as shown in Figure 4. The achieved values of PCE cost function in the cases of EPSO, PSO, and Bone et al. are 3.19*E* + 2, 2.77*E* + 2, and 2.72*E* + 1, respectively. The obtained results of EPSO based on PCE cost function again outmatch the results obtained for PSO and Bone et al.'s proposed algorithm. The obtained optimized values clearly depict a sharper peak in the case of EPSO as compared with PSO and Bone et al.

Figure 5 shows a 15° out of plane rotated testing image. The optimized values generated from EPSO are yielding much sharper peaks as compared to the optimized values generated through PSO or the conventional values of Bone et al.'s algorithm. The PCE values for 15° out of plane rotated testing image for EPSO, PSO, and Bone et al. are 5.01*E* + 2, 5.72*E* + 1, and 3.92*E* + 1. The results obtained by using conventional PSO are better than the results obtained from Bone et al.'s algorithm. However, the EPSO-generated optimized values give the best results as compared to the results obtained from the optimized values generated from PSO and Bone et al., in terms of PCE and COPI cost functions. The optimized values depend on the images contained in the dataset. The cost functions and the datasets define the values of the optimized parameters.

The article "Optimization of Correlation Filters Using Extended Particle Swarm Optimization Technique" was retracted in 2023. Reasons: unreliable results or conclusions; concerns about the data; concerns about the peer review; concerns about the citations.

## 4. Conclusion

A novel technique has been proposed which combines optimization algorithms with a correlation filter in order to improve the results of the correlation filter. The technique focuses on optimizing the tradeoff parameters pertaining to correlation filters which have not been achieved earlier. The optimization parameters achieved by using EPSO and PSO algorithms have been compared with the optimization values of the previously employed algorithms. The comparison was based on the PCE and COPI cost functions for a specific object recognition application. The values are not constant for all the object recognition applications as suggested by the previous studies. The values of optimal tradeoff parameters and the PCE and COPI cost functions are calculated for specific datasets based on their properties. The EPSO optimized values helped in the reduction of the ONV factor thus resulting in more accurate results as compared to the PSO and other previously suggested similar algorithms. The proposed work also has plenty of scope for future studies. In the future, we will try to compare EPSO and PSO with more advanced heuristic algorithms in order to achieve more accurate results. A few recent algorithms are improved GA, grasshopper, mothflame, and name a few more [37–39].

## Figures and Tables

**Figure 1:** Datasets.

**Figure 2:** (a) Correlation plane using Bone et al. values, (b) PSO value-based correlation plane, (c) ESPO correlation plane values, and (d) testing image.

**Figure 3:** (a) Bone et al. value-based correlation plane, (b) PSO value-based correlation plane, (c) ESPO correlation plane values, and (d) testing image.

**Figure 4:** (a) Correlation plane using Bone et al. values, (b) PSO value-based correlation plane, (c) ESPO correlation plane values, and (d) testing image.

**Figure 5:** (a) Bone et al. value-based correlation plane, (b) PSO value-based correlation plane, (c) ESPO correlation plane values, and (d) testing image.

**Table 1:** Parameter optimization of correlation filter using PSO.

	Optimal tradeoff parameter estimation for correlation filter using PSO
1.	Each particle's position and velocity parameters are randomly initialized
2.	Fitness function value estimation using Equations (15) and (17) for each particle
3.	Calculation of best value for each particle
4.	Calculation of Swarm's global best
5.	The position of particles is updated using Equation (11) [19]
6.	The velocity of particles is updated using Equation (10) [19]
7.	Fitness function value estimation using Equations (16) and (17) for each particle
8.	Calculation of local best pertaining to each particle
9.	Calculation of global best pertaining to each swarm
10.	If stopping condition is achieved, terminate the algorithm. Otherwise, go back to Step 5

The article "Optimization of Correlation Filters Using Extended Particle Swarm Optimization Technique" was retracted in 2023. Reasons: unreliable results or conclusions; concerns about the data; concerns about the peer review; concerns about the citations.

**Table 2:** Parameter optimization of correlation filter using EPSO.

	Optimal tradeoff parameter estimation for correlation filter using EPSO
1.	Each particle's position and velocity parameters are randomly initialized
2.	Fitness function value estimation using Equations (16) and (17) for each particle
3.	Calculation of local best pertaining to each involved particle
4.	Calculation of global best pertaining to each involved swarm
5.	The position of particles is updated using Equation (15) [21]
6.	The velocity of particles is updated using Equation (17) [21]
7.	Reinitialize the velocity if the velocity of particles becomes equal to zero
8.	Fitness function value estimation using Equations (16) and (17) for each particle
9.	Calculation of local best pertaining to each particle
10.	Calculation of global best pertaining to each swarm
11.	If stopping condition is achieved, terminate the algorithm. Otherwise, go back to Step 5

**Table 3:** Setting of PSO parameter values.

Parameter setting	Values
Experiments	120
Iterations	320
Particles	10
Dimensions	03
*X*_min_	-1
*X*_max_	1
*V*_min_	-0.1
*V*_max_	0.1
*W*	0.9
*C*_1_, *C*_2_	2

**Table 4:** COPI value comparison.

Dataset	Testing image (degree)	Bone et al. values (COPI)	PSO				EPSO			
			*α*	*β*	*γ*	COPI	*α*	*β*	*γ*	COPI
1	5	4.05*E* − 5	0.0040	0.0402	0.0473	2.74*E* − 4	8.45*E* − 9	0.0954	0.1722	2.74*E* − 1
2	5	4.91*E* − 5	0.0040	0.0421	0.0506	3.91*E* − 4	7.39*E* − 9	0.0921	0.2102	2.04*E* − 1
3	15	2.05*E* − 5	0.0041	0.0404	0.0470	6.05*E* − 5	3.04*E* − 8	0.0726	0.2232	1.24*E* − 1
4	15	3.98*E* − 5	0.0038	0.0388	0.0525	1.98*E* − 3	2.14*E* − 8	0.1229	0.2212	1.37*E* − 0
5	25	4.15*E* − 5	0.0035	0.0389	0.0499	3.15*E* − 4	1.45*E* − 8	0.1021	0.1639	1.34*E* − 1
6	25	5.05*E* − 5	0.0039	0.0384	0.0473	4.01*E* − 4	8.45*E* − 8	0.1512	0.1978	1.74*E* − 1
7	45	4.95*E* − 5	0.0042	0.0310	0.0428	3.15*E* − 4	6.27*E* − 9	0.2102	0.1099	2.44*E* − 2
8	45	7.05*E* − 5	0.0039	0.0390	0.0478	5.15*E* − 4	7.45*E* − 9	0.1022	0.1877	3.24*E* − 2

**Table 5:** Comparison of PCE values for EPSO, PSO, and Bone et al.'s values.

Dataset	Testing image (Deg.)	Bones values (PCE)	PSO				EPSO			
			*α*	*β*	*γ*	PCE	*α*	*β*	*γ*	PCE
1	5	6.02*E* + 1	0.0034	0.7232	0.5449	1.62*E* + 2	2.19*E* − 6	0.7134	0.4772	7.74*E* + 2
2	5	5.14*E* + 1	0.0040	0.7492	0.5781	7.52*E* + 1	1.35*E* − 6	0.7293	0.4923	6.34*E* + 2
3	15	4.95*E* + 1	0.0029	0.7321	0.5322	1.62*E* + 2	1.72*E* − 5	0.7522	0.3982	8.04*E* + 2
4	15	3.92*E* + 1	0.0039	0.7002	0.5349	5.72*E* + 1	4.83*E* − 8	0.6578	0.4438	5.01*E* + 2
5	25	4.32*E* + 1	0.0031	0.7244	0.5449	2.69*E* + 2	2.44*E* − 7	0.7980	0.5223	2.74*E* + 3
6	25	1.48*E* + 2	0.0032	0.7390	0.5019	1.42*E* + 2	7.19*E* − 7	0.6991	0.4938	2.14*E* + 3
7	45	2.72*E* + 1	0.0034	0.7470	0.5709	2.77*E* + 2	4.19*E* − 7	0.5224	0.6220	3.19*E* + 2
8	45	3.24*E* + 1	0.0030	0.6295	0.5014	1.99*E* + 2	3.59*E* − 7	0.4900	0.5114	2.44*E* + 2

The article "Optimization of Correlation Filters Using Extended Particle Swarm Optimization Technique" was retracted in 2023. Reasons: unreliable results or conclusions; concerns about the data; concerns about the peer review; concerns about the citations.

## Data Availability

The imaging data used to support the findings of this study are included within the article.
